# Activation of Neural Modeling-Related Genes in the Heart of Mice after Gamma Irradiation

This article has been retracted.

**DOI:** 10.1155/2021/8522417

**Published:** 2021-12-31

**Authors:** Zhiyong Liu, Jing Liu, Dan Hu, Juanjuan Du, Donglu Liu, Ximin Wang, Jiandong Zhang, Yinglong Hou

**Affiliations:** ^1^Department of Cardiology, Shandong Qianfoshan Hospital, Cheeloo College of Medicine, Shandong University, Jinan, Shandong 250012, China; ^2^Department of Cardiology, Dezhou People's Hospital, Dezhou, Shandong 253014, China; ^3^Department of Endocrinology, Dezhou People's Hospital, Dezhou, Shandong 253014, China; ^4^Department of Oncology, The First Affiliated Hospital of Shandong First Medical University & Shandong Provincial Qianfoshan Hospital, Jinan, Shandong 250012, China; ^5^Cheeloo College of Medicine, Shandong University, Jinan, Shandong 250012, China

## Abstract

**Objective:**

Radiation-induced heart disease (RIHD) is a common sequela of thoracic irradiation. At the same time, nerve remodeling is involved in the progression of heart disease. However, the activation of the nerve remodeling related genes in radiation-induced heart disease is still lacking.

**Methods:**

In this study, C57BL/J mice was anesthetized by intraperitoneal injection with pentobarbital sodium (2%, 40 mg/kg), and radiation was delivered using a cobalt-60 (^60^Co) teletherapy unit (Cirus). When the mice were anesthetized, none of them showed the signs of peritonitis, pain, or discomfort. The mice hearts were exposed to a *γ*-radiation field of 5 mm × 5 mm. The total dose of *γ*-radiation was 3 Gy/day for each animal for 5 consecutive days. The mice were executed by severed neck, and its limbs were weak. Quantitative Polymerase Chain Reaction (qPCR) and immunohistochemistry were used to explore the possible mechanism of arrhythmia in patients with RIHD.

**Results:**

Our results demonstrated that Growth-Associated Protein 43 (GAP43) was increased significantly after radioactive heart injury compared with the control group. Moreover, the protein expression of Tyrosine hydroxylase (TH) and Choline acetyl-transferase (CHAT) was significantly decreased compared with the control group and gradually increased with time rend. The nerve growth factor (NGF) was remarkably increased after radiation-induced heart injury compared with the control group. Immunohistochemistry results indicated that the nerve growth factors GAP43 and NGF were significantly increased after radiation-induced heart injury.

**Conclusions:**

Chest radiotherapy could activate the neural modeling related genes in RIHD. This may provide a new treatment plan for the future treatment of heart problems caused by chest radiotherapy.

## 1. Introduction

Radiotherapy is an indispensable part of multidisciplinary treatment of malignancies. It has previously been proposed that approximately 52.3% of all oncological patients should receive radiation during the course of their illness [1]. Normal tissue injury associated with radiotherapy is clinical issues of multidisciplinary treatment for malignancies. Radiation-induced heart diseases (RIHDs) have become one of the major causes of nonneoplastic death in patients receiving thoracic irradiation, especially with old technique of radiotherapy, particularly in patients with classical Hodgkin's lymphoma [2–4] and early-stage breast cancer [5–7]. The application of more sophisticated techniques has greatly decreased the dose delivered to the whole heart and its substructures. Nevertheless, cardiac toxicity remains a major concern when balancing target coverage and minimizing cardiac dose in delivering radiotherapy to thoracic tumors. Some patients have shown that cardiovascular morbidity was increased in several years after IR, with acute and chronic effects of RIHDs [8]. The cardiovascular complications of radiotherapy are generally coronary artery disease, pericardial disease, cardiomyopathy/myocardial fibrosis, valvular disease, and arrhythmia [9].

The previous study has reported that patients have an increased risk of ventricular tachyarrhythmia and sudden cardiac death (SCD) [10–12] and increased sympathetic nerve density is the occurrence of lethal arrhythmias [13]. The mechanisms of neural remodeling have been studied extensively [14, 15]. Growing evidence showed that inflammation and its associated cytokines can play a key role in stimulating neurite growth and regeneration.

More and more studies have found that some heart diseases will be accompanied by different nerve density, promoting the occurrence of arrhythmias, such as ventricular and atrial arrhythmias [16–18]. Researchers hope to find a more appropriate intervention to reduce arrhythmia caused by cardiac nerve remodeling through in-depth research on the phenomenon of cardiac nerve remodeling and its relationship with arrhythmia. Because the heart nerve is plastic, when the nerve is injured, it will be denervated, with nerve eruption and excessive regeneration [15, 19, 20]. At present, the mechanism of cardiac nerve sprouting and excessive regeneration is not clear, but the role of nerve growth factor in nerve remodeling is self-evident [21, 22].

Nerve remodeling has different regulatory functions in different diseases. For example, in Alzheimer's disease, nerve remodeling is beneficial to the development of brain nerves and promotes nerve regeneration, but in heart diseases, nerve remodeling leads to arrhythmia and other problems. Therefore, for the function of nerve remodeling, different disease types have different functions.

The nerve remodeling of the heart refers to the function adjustment of the autonomic nerves of the heart. The autonomic nervous system of the heart is divided into the external cardiac autonomic nervous system and the internal cardiac autonomic nervous system. The external cardiac autonomic nerve includes the sympathetic nervous system and the parasympathetic nervous system. The sympathetic nerve fibers mainly come from the cervical spine C1-3 and the thoracic vertebra C7-8 T1-2 spinal ganglia; anatomically, the external cardiac autonomic nervous system refers to the connection between the heart and the brain or the nerve fibers of the spinal cord. In addition to the external cardiac autonomic nervous system, there is also an exquisite and perfect internal cardiac autonomic nervous system. The inner cardiac autonomic nervous system refers to a large number of ganglia throughout the heart, each ganglion contains 200 to 1000 neurons, and the sympathetic and parasympathetic nerve fibers in the pericardial cavity form synaptic connections.

NGF is one of the body's important neurotrophic factors. Nerve remodeling can be observed by increasing the expression of NGF in the heart after myocardial infarction. The function of NGF inhibition could reduce the growth of sympathetic nerve in myocardial infarction tissue [23]. In some heart diseases, neural remodeling has a bad effect, such as causing ventricular arrhythmias and sudden death. In addition, the density of nerve fibers was increased significantly after myocardial infarction, and the induction rate of ventricular arrhythmia also was increased correspondingly [23]. Clinical studies have shown that both the sympathetic and parasympathetic nervous systems can promote atrial arrhythmias [24].

TH is a rate-limiting enzyme that it can catalyze the synthesis of catecholamine neurotransmitters. It is abundantly expressed in sympathetic ganglia and sympathetic norepinephrine neurons, and its positive expression can reflect the distribution of sympathetic nerves in the heart [25]. CHAT is a specific marker enzyme of cholinease, which reflects the distribution of vagus nerve in the heart [26]. GAP43 is a fast-transporting membrane phosphoprotein expressed in the growth mound of budding axons. It was widely distributed in autonomic neurons and is closely related to nerve development, axon regeneration, synaptic reconstruction, and transmitter release. It is an intrinsic determinant of neuron development and regeneration. Its existence marks the growth of nerves and can be used to evaluate the growth activity of autonomic nerves. TH, CHAT, and GAP43 are the main markers of cardiac autonomic nerves, and their expression level can be used as an important basis for autonomic nerve regeneration.

In this study, the transcription and protein expression of genes related to nerve remodeling after chest radiotherapy were detected by RT-qPCR and tissue immunohistochemical experiments. Subsequently, biochemical indicators were detected to explore the heart disease caused by chest radiotherapy. The problem of nerve remodeling provides a scientific basis for the future treatment of nerve remodeling in heart disease.

## 2. Materials and Methods

### 2.1. Ethical Statement

The study was approved by the Ethics Committee of Cheeloo College of Medicine, Shandong University (No. S026). Moreover, we follow the principles on ethical animal research outlined in the Basel Declaration and the ethical guidelines by the International Council for Laboratory Animal Science (ICLAS).

### 2.2. Clinical Case Materials

We selected 180 lung cancer patients who underwent IMRT at Dezhou People's Hospital from January 2018 to December 2019, of which 102 were males and 78 were females; they were 41 to 72 (51.37 ± 10.01) years old. The following are the inclusion criteria: patients met the pathological and histological diagnostic criteria of lung cancer; the lesion is located in the left lung; and all patients received intensity-modulated radiotherapy. The following are the exclusion criteria: patients with other malignant tumors and patients with severe mental illness. The study was approved by the ethics committee of our hospital, and the patients and their families were aware of the specific content of the study and signed an informed consent form.

### 2.3. Animals and Irradiation Exposure Protocol

Male C57BL/J mice (10-week-old) provided by the Animal Experimental Centre of Shandong University were used in this study. Animals were raised in isolated cages in temperature-controlled rooms and were provided continuous 12 h artificial dark-light cycles. Animals received standard mouse chow and had free access to tap water. The irradiation protocol was implemented in accordance with descriptions in previous reports but with some modifications [16]. Mice were anesthetized by intraperitoneally injection with pentobarbital sodium (2%, 40 mg/kg), and radiation was delivered using a cobalt-60 (^60^Co) teletherapy unit (Cirus). When the mice were anesthetized, none of them showed signs of peritonitis, pain, or discomfort. The mouse hearts were exposed to a *γ*-radiation field of 5 mm × 5 mm. The total dose of *γ*-radiation was 15 Gy. The specific details are 3 Gy/day for each animal for 5 consecutive days. After the last exposure, the mice were immediately executed by severed neck, and its limbs were weak to prove that it was completely executed.

### 2.4. Experimental Design

Twenty experimental mice (C57BL/J) were divided evenly and randomly into 10 irradiated mice and 10 unirradiated controls (Ctrl).

### 2.5. RNA Extraction and Quantitative RT-PCR

Total RNA was extracted from the heart tissue and reverse transcribed into cDNA by SuperScript III Reverse Transcriptase (Invitrogen, Grand Island, NY, USA) according to a protocol. Quantitative real-time PCR was performed in the CFX96 PCR system. The PCR amplification conditions were as follows: 95°C for 10 min, followed by 40 cycles of 95°C for 10 s and 60°C for 1 min. The relative levels of mRNA were calculated using the 2^-*ΔΔ*Ct^ method and normalized to *β*-actin.

### 2.6. Immunohistochemistry

Sections were incubated with 3% H_2_O_2_ for 15 min, then blocked with goat serum protein (Solarbio, Beijing, China) for 30 min at 37°C. After pouring slowly, it was incubated with the corresponding primary antibody overnight at 4°C. The primary antibody was presented as follows: rabbit polyclonal to NGF (1 : 1000; ab6199, Abcam, Cambridge, MA, USA), TH (1 : 800; ab6211, Abcam), CHAT (1 : 1000; ab6168, Abcam), and GAP43 (1 : 1000; ab16053, Abcam). After incubation at 37°C for 1 h and washing with 0.1 M PBS three times, secondary antibodies (1 : 3000; Abcam) were added to incubate for 20 min. After washing sections, it was visualized using the DAB reagent. Nuclear counter stain hematoxylin was dehydrated with ethanol and mounted with glycerol gelatin. Images were measured using ImageJ 6.0 system.

### 2.7. Statistical Analysis

Data collected in this study were expressed as the mean ± SD. The data were analysed using the SPSS software (v.20.0, SPSS) using Student's *t*-tests. A *P* value < 0.05 was considered statistically significant.

## 3. Results

### 3.1. Data of Arrhythmia after Intensity-Modulated Radiotherapy for Malignant Lung Tumors

Compared with before radiotherapy, the ECG at 6 weeks after radiotherapy, sinus arrhythmia was significantly increased, which was statistically significant (*P* < 0.05); compared with before radiotherapy, occasional atrial (ventricular) arrhythmia occurred at 6 weeks after radiotherapy The changes of ST-T segment increased significantly, with a statistical difference (*P* < 0.01); compared with before radiotherapy, 6 weeks after radiotherapy, conduction block radiation increased significantly, which was statistically significant (*P* < 0.01); compared with before radiotherapy, the ECG of frequent atrial (ventricular) arrhythmia increased significantly after 6 weeks of radiotherapy, with statistical difference (*P* < 0.01) (see Table 1).

### 3.2. Nerve Growth Factor GAP43 and NGF mRNA Expression Were Increased after Gamma Irradiation

Growth-associated protein 43 (GAP43) can be used as a marker for nerve sprouting. Studies have shown that nerve growth factor (NGF) synthesized and released by damaged myocardium and inflammatory tissue plays an important role in nerve remodeling. Therefore, changes in GAP43 and NGF indicators can reflect changes in nerves. As illustrated in Figure 1, the GAP43 and NGF mRNA expression in tissue samples of the RIHD mice was higher than that of normal mice (*P* < 0.001) by RT-qPCR. These results demonstrated that radiation heart injury will lead to changes in nerve-related factors.

### 3.3. Nerve Growth Factor GAP43 and NGF Protein Expression Were Increased after Gamma Irradiation

As the previous experiments found that the transcription levels of GAF43 and NGF increased significantly, we wanted to observe whether the levels of GAF43 and NGF proteins also changed in the same trend, so immunohistochemistry experiments were used to detect the expression of GAF43 and NGF proteins. As illustrated in Figure 2, the GAP43 and NGF protein expression in tissues samples of the RIHD mice was higher than that of normal mice (*P* < 0.05) by immunohistochemistry. These results demonstrated that radiation heart injury will lead to changes in nerve-related factors.

### 3.4. TH and CHAT Protein Expression Were Increased after Gamma Irradiation

We all know that TH and CHAT are two marker molecules for nerve fibers, so in this study, we tested these two indicators. As illustrated in Figure 3, the TH and CHAT protein expression in tissues samples of the RIHD mice was higher than that of normal mice (*P* < 0.05) by immunohistochemistry.

## 4. Discussion

Radiotherapy is an indispensable part of the comprehensive treatment of malignant tumors. When esophageal cancer, lung cancer, breast cancer, mediastinal lymphoma and other tumor tissues received the radiotherapy, the heart adjacent to the tumor tissue will also be irradiated with different dose and volumes. Radiation-induced heart disease (RIHD) may or may not cause clinical symptoms. However, radiation can destroy vascular endothelial cells and microcirculation system, which in turn can cause ischemic changes in myocardium and ultimately lead to damage to the structure and function of the heart [19]. Although due to the advancement of radiotherapy technology and other factors, the radiation dose of the heart has been greatly reduced, the damage to the heart by radiation cannot be ignored [26]. At present, there is no clear consensus on the prevention and treatment of RIHD. Therefore, how we simulate and construct experimental animal models of RIHD with clinical symptoms and then reveal the possible mechanism of radiation heart injury is of great significance for the prevention and treatment of RIHD. A previous literature reported that the heart would suffer irreversible damage after exposure to a single dose of 3 Gy. Therefore, this experiment constructs a model by observing the characteristics of different damage caused by different doses of radiation and provides a scientific and feasible animal model for the next experiment.

In this study, we used real-time fluorescent quantitative PCR and immunohistochemistry to study the expression of TH, CHAT, and GAP43 at the mRNA and protein. The results showed that compared with the control group, the expression levels of mRNA and protein of TH, CHAT, and GAP43 in the heart tissue of the radiation heart injury group were increased significantly. This study was the first to test the expression levels of positive markers representing sympathetic and vagal nerve fibers in the cardiac tissue. It was found that TH, CHAT, and GAP43 were significantly increased, suggesting that both sympathetic and vagal nerves may be involved in the triggering and maintenance of arrhythmia. The specific triggering and maintenance of arrhythmia and its relationship have not yet been fully elucidated.

Cardiac autonomic nerve and arrhythmia are mutually causal. In the increase and uneven distribution of cardiac autonomic nerves affect the electrophysiological characteristics of the atrial, which in turn leads to the occurrence and maintenance of atrial electrical remodeling and arrhythmia. Persistent arrhythmia can lead to atrial enlargement and insufficient blood supply. Structural remodeling leads to myocardial damage, which in turn causes nerve damage. The development and repair of nerves by GAP43 regenerate damaged nerves, which also promotes the growth of undamaged nerves in the increased abd uneven. Therefore, in the process of sympathetic nerve reconstruction, as the vagus nerve is rebuilt, arrhythmia causes myocardial ischemia, and neurohormones such as elevated levels of cytokines and growth factors in the circulation may be the cause of atrial nerve growth.

In conclusion, our results revealed that chest radiotherapy could activate the neural modeling-related genes in RIHD. This may provide a new treatment plan for the future treatment of heart problems caused by chest radiotherapy.

## Figures and Tables

**Figure 1:** Nerve growth factor GAP43 and NGF mRNA expression was increased after radiation heart injury. ^∗∗∗^*P* < 0.001.

**Figure 2:** Nerve growth factor GAP43 and NGF protein expression was increased after radiation heart injury. ^∗^*P* < 0.05. The yellowish-brown blot represents a positive signal.

**Figure 3:** TH and CHAT protein expression was increased after radiation heart injury. ^∗^*P* < 0.05. The yellowish-brown blot represents a positive signal.

**Table 1:** Basic information of the patient's 24 h ambulatory electrocardiogram (*n*(%), *n* = 180).

Time	Sinus arrhythmia	Occasional atrial (ventricular) arrhythmia	Frequent atrial (ventricular) arrhythmia	Conduction block	ST-T segment changes
Before the start of the treatment	33 (16.5)	61 (30.5)	45 (22.5)	21 (10.5)	29 (14.5)
End of the treatment	52 (26.0)	109 (54.5)	79 (39.5)	38 (19.0)	71 (35.5)
6 weeks after the end of the treatment	47 (23.5^∗^)	96 (48.0^∗∗^)	71 (35.5^∗∗^)	30 (15.0^∗^)	36 (18.0^∗^)

Compared with before radiotherapy, ^∗^*P* < 0.05 and ^∗∗^*P* < 0.01.

## Data Availability

The data used to support the findings of this study are available from the corresponding author upon request.
